# Heat Shock Cognate 70 Inhibitor, VER-155008, Reduces Memory Deficits and Axonal Degeneration in a Mouse Model of Alzheimer’s Disease

**DOI:** 10.3389/fphar.2018.00048

**Published:** 2018-01-30

**Authors:** Ximeng Yang, Chihiro Tohda

**Affiliations:** Division of Neuromedical Science, Department of Bioscience, Institute of Natural Medicine, University of Toyama, Toyama, Japan

**Keywords:** Alzheimer’s disease, Heat shock cognate 70, axonal regeneration, memory recovery, VER-155008, 5XFAD mice

## Abstract

Alzheimer’s disease (AD) is a progressive neurodegenerative disorder resulting in structural brain changes and memory impairment. We hypothesized that reconstructing neural networks is essential for memory recovery in AD. Heat shock cognate 70 (HSC70), a member of the heat shock protein family of molecular chaperones, is upregulated in AD patient brains, and recent studies have demonstrated that HSC70 facilitates axonal degeneration and pathological progression in AD. However, the direct effects of HSC70 inhibition on axonal development and memory function have never been investigated. In this study, we examined the effects of a small-molecule HSC70 inhibitor, VER-155008, on axonal morphology and memory function in a mouse model of AD (5XFAD mice). We found that VER-155008 significantly promoted axonal regrowth in amyloid β-treated neurons *in vitro* and improved object recognition, location, and episodic-like memory in 5XFAD mice. Furthermore, VER-155008 penetrated into the brain after intraperitoneal administration, suggesting that VER-155008 acts in the brain *in situ*. Immunohistochemistry revealed that VER-155008 reduced bulb-like axonal swelling in the amyloid plaques in the perirhinal cortex and CA1 in 5XFAD mice, indicating that VER-155008 also reverses axonal degeneration *in vivo*. Moreover, the two main pathological features of AD, amyloid plaques and paired helical filament tau accumulation, were reduced by VER-155008 administration in 5XFAD mice. This is the first report to show that the inhibition of HSC70 function may be critical for axonal regeneration and AD-like symptom reversal. Our study provides evidence that HSC70 can be used as a new therapeutic target for AD treatment.

## Introduction

Deposits of amyloid β (Aβ) and hyperphosphorylated tau in the brain are the two main pathological features of Alzheimer’s disease (AD). These deposits trigger the disruption of neural networks in the brain, which is the direct cause of memory dysfunction in AD. Reconstruction of damaged neural networks, including neurite regeneration and synapse re-formation, may be essential for memory function recovery. New drugs and new therapeutic targets that prevent or reverse axonal degeneration are needed to preserve memory function in AD.

Heat shock cognate protein 70 (HSC70) is a molecular chaperone from the heat shock protein (HSP) family (Stricher et al., 2013). Multiple intracellular functions of HSC70 have been reported, including binding and promoting the folding of nascent polypeptides, degrading client proteins via the ubiquitin proteasome system (UPS) (Meimaridou et al., 2009), and chaperone-mediated autophagy (CMA) (Cuervo, 2011). HSC70 expression is increased in AD model mice and patient brains (Piedrahita et al., 2016), and HSC70 prevents the accumulation of phosphorylated tau (Jinwal et al., 2010). Importantly, neurofilament medium chain protein (NF-M), a component of neurites, interacts with HSC70 and is degraded by the UPS (Wang et al., 2011), possibly facilitating axonal degeneration in AD. Therefore, HSC70 upregulation in AD brains might contribute to memory deficits. However, no reports have demonstrated a direct effect of HSC70 inhibition on axonal development or memory function.

The 5XFAD (Tg6799) AD mouse model co-expresses mutant human amyloid precursor protein (APP) containing the Swedish (K670N and M671L), Florida (I716V), and London (V717I) mutations, and presenilin-1 (PS1; M146L and L286V) specifically in neurons. These five familial AD mutations increase the level of Aβ_1-42_ peptide in the brain (Oakley et al., 2006). Aβ plaques deposition begins at 2 months, and memory deficit is first observed at 4 months of age in 5XFAD mice.

VER-155008 is an HSC70 functional inhibitor that competitively binds to the ATP-binding pocket of HSC70 (Schlecht et al., 2013). Approximately 10 small-molecule inhibitors of HSC70 are known (Goloudina et al., 2012); however, it is difficult to isolate the specific inhibitory effect on HSC70 because of its sequence similarity to other HSPs (86% for HSP70). We selected VER-155008 because of its sustained inhibitory effect on HSC70 but not HSP70 (Schlecht et al., 2013).

In the present study, we investigated the effects of HSC70 inhibition by VER-155008 on axonal development in cultured neurons and memory function in 5XFAD mice. We also examined the pathological changes in the brain tissue of VER-155008-treated 5XFAD mice. The goal of this study was to evaluate HSC70 function inhibition as a potential strategy for treatment of AD.

## Materials and Methods

All experiments were performed in accordance with the Guidelines for the Care and Use of Laboratory Animals of the University of Toyama. The Committee for Animal Care and Use at the Sugitani Campus of the University of Toyama approved the study protocols (approval number for the animal experiments is A2017INM-1). All efforts were made to minimize the number of animals used.

### Animal Studies

Transgenic mice (5XFAD) were obtained from the Jackson Laboratory (Bar Harbor, ME, United States) and maintained by crossing hemizygous animals with B6/SJL F1 breeders. To investigate the effect of VER-155008 on 5XFAD mice, we used hemizygous female mice (age: 32–38 weeks in the experiments shown in **Figures 2A–D**, and 24–28 weeks old in **Figures 2E–H**) or wild-type female littermates. All mice were housed with free access to food and water in a controlled environment (22 ± 2°C, 12 h light/dark cycle starting at 7:00 am).

### Behavioral Tests

To investigate the relationship between HSC70 inhibition and memory recovery, VER-155008 (IC_50_ = 0.5 μM; Sigma–Aldrich, St. Louis, MO, United States) was dissolved in 10% dimethyl sulfoxide (DMSO)-containing saline and administered intraperitoneally (10 μmol/kg/day) to 5XFAD mice for 18 days (**Figures 2A–D**) or 15 days (**Figures 2E–H**). Vehicle solution (10% DMSO in saline) was used as a control. On day 14 of administration, the novel object recognition or location test and on day 15, the episodic-like memory test were performed as described previously (Kuboyama et al., 2015). Testing was performed in a dimly illuminated (81 lux) room. On the last day of administration, mice were individually habituated to an open-field box composed of polyvinyl chloride (33 cm × 29 cm; height, 26.5 cm) for 10 min. Their paths were tracked using a digital camera system. The total distance moved (cm) and total immobility time (s) for 10 min were analyzed with EthoVision 3.0 (Noldus, Wageningen, Netherlands).

### Brain Penetration of VER-155008

To detect the blood brain barrier (BBB) penetration, VER-155008 or vehicle solution (10% DMSO in saline) was intraperitoneally administered (89.9 μmol/kg) to female 5XFAD mice (36 weeks old). Five minutes after drug administration, the mice were euthanized by isoflurane and blood was collected. The plasma was obtained after centrifugation at 10,000 *g* for 10 min at 4°C. Plasma (120 μl) was extracted with methanol, dried, and resolubilized in 100 μl of methanol. The cerebral cortex perfused with saline before dissection was homogenized, extracted with methanol, dried, and resolubilized in 100 μl of methanol before LC-MS analysis. To calculate the VER-155008 concentration in the cortex, a standard curve was plotted. Briefly, standard solutions of VER-155008 were mixed with a control cortex extract, prepared as the above, and subjected to LC-MS analyses. A Thermo Scientific^TM^ Accela HPLC system interfaced with an LTQ Orbitrap XL hybrid Fourier Transform Mass Spectrometer (Thermo Fisher Co., San Jose, CA, United States) was used to chemically profile VER-155008. Liquid chromatographic analyses were performed on a Capcell Pak C18 MGIII S-5 (1.5 mm i.d. × 150 mm, Shiseido, Tokyo, Japan) column held at 40°C with a flow rate of 200 μl/min. Ultrapure water and ethanol (E) were used as the mobile phase. The following linear elution gradient was used: 0–5 min, 40–70% E; 5–10 min, 70–85% E; 10–13 min, 85–100% E; 13–14 min, 100–40% E; 14–18 min, 40% E. The following electrospray ionization (ESI) parameters were used: spray voltage, 4.5 kV; capillary voltage, 40.0 kV; tube lens, 150 V; capillary temperature, 330°C; sheath gas flow rate, 50 units; and aux gas flow rate, 10 units. We operated the mass spectrometer in the positive ESI mode; scanning from 50 to 2,000 m/z; and calibrated the instrument using a polytyrosine solution before each experiment.

### Primary Culture and Immunocytochemistry

Embryos were removed from a pregnant ddY mouse (Japan SLC, Shizuoka, Japan) at 14 days of gestation as described previously (Tohda et al., 2012). Cells were treated with or without 10 μM Aβ_25-35_ (Sigma–Aldrich) for 3 days, followed by the addition of 0.05, 0.5, or 5 μM VER-155008 or vehicle solution (0.1% DMSO) for 4 days. The Aβ_25-35_ was incubated at 37°C for 4 days prior to treatment to facilitate aggregation. The cells were fixed with 4% paraformaldehyde and immunostained at 4°C for 24 h with antibodies against the axonal marker, mouse phosphorylated neurofilament heavy subunit (pNF-H; monoclonal, 1:250, Covance, Princeton, NJ, United States), and against the neuronal marker, rabbit microtubule-associated protein 2 (polyclonal, 1:3000, Abcam, Cambridge, United Kingdom). Alexa Fluor 488-conjugated goat anti-mouse IgG (1:400) and Alexa Fluor 568-conjugated goat anti-rabbit IgG (1:400) were used as secondary antibodies. Fluorescence images (864.98 μm × 645.62 μm) were captured using a fluorescence microscopy system (Carl Zeiss, Oberkochen, Germany). The lengths of the pNF-H-positive axons were measured using MetaMorph version 7.8 (Molecular Devices, Sunnyvale, CA, United States).

### Immunohistochemistry

After behavioral tests, mice were deeply anesthetized by 30 mg/ml chloral hydrate and perfused with ice-cold saline. The brains were carefully removed from the skull, immersed in ice-cold 4% paraformaldehyde for 24 h at 4°C, immersed in 30% sucrose for 7 days for cryoprotection, and stored at -30°C. The brains were cut into 20 μm coronal slices every 100 μm in the perirhinal cortex area (bregma -1.46 to -2.06 mm) using a cryostat (Leica, Heidelberg, Germany). The slices were fixed with 4% paraformaldehyde and immunostained at 4°C for 24 h with an antibody against rabbit Aβ(1-40/42) (polyclonal, 1:400, Chemicon, Temecula, CA, United States) and an antibody against mouse pNF-H (monoclonal, 1:500, Covance) or against mouse paired helical filament (PHF)-tau (pSer202+Thr205; AT8) (monoclonal, 1:100, Thermo Scientific, Rockford, IL, United States). Alexa Fluor 568-conjugated goat anti-rabbit IgG (1:400) and Alexa Fluor 488-conjugated goat anti-mouse IgG (1:400) were used as secondary antibodies. Staining with 1 μg/ml DAPI (4′, 6-diamidino-2-phenylindole) was performed at room temperature for 10 min. Fluorescence images (864.98 μm × 645.62 μm) were captured using a fluorescence microscope (BX-61/DP70, Olympus, Tokyo, Japan). Six to eight successive brain slices of the perirhinal cortex of each mouse were captured for quantification. The images were analyzed using the image analysis software, ImageJ as described previously (Tohda et al., 2012).

### Statistical Analysis

Statistical comparisons were performed using one-way analysis of variance (ANOVA) with *post hoc* Dunnett’s tests, repeated measures two-way ANOVA with the *post hoc* Bonferroni test, and unpaired *t*-tests in GraphPad Prism 5 (GraphPad Software, La Jolla, CA, United States). *p* < 0.05 was considered significant. Data are presented as the mean ± standard deviation.

## Results

### VER-155008 Reverses Aβ-induced Axonal Atrophy in Cultured Neurons

To investigate the effect of HSC70 inhibition on axonal morphology, Aβ-treated neurons were further treated with VER-155008. After 3 days of Aβ (10 μM) treatment, the length of the pNF-H-positive axons was significantly reduced. However, a subsequent addition of 0.05–5 μM VER-155008, but not vehicle, restored the axonal length to the control levels (**Figure 1**). This result suggests that the inhibition of HSC70 function can induce axonal regrowth after Aβ treatment of neurons.

**FIGURE 1:** VER-155008 treatment reversed Aβ-induced axonal degeneration in cultured neurons. Mouse cortical neurons (ddY, E14) were cultured for 3 days and then treated with or without Aβ_25-35_ (10 μM) for another 3 days. After the 3 days of Aβ_25-35_ treatment, the neurons were treated with VER-155008 (0.05, 0.5, or 5 μM) or vehicle solution (0.1% DMSO) for 4 days, fixed and immunostained for phosphorylated neurofilament heavy subunit (pNF-H). **(A)** Representative images of pNF-H-positive axons from each treatment are shown. **(B)** Lengths of pNF-H-positive axons were quantified in each treatment group. ^∗∗^*p* < 0.01, ^∗∗∗^*p* < 0.001 vs. Aβ_25-35_/Veh, one-way ANOVA *post hoc* Dunnett’s test. The number of measured areas is shown in each column.

### VER-155008 Improves Memory Function in 5XFAD Mice

Next, to investigate the relationship between the inhibition of HSC70 and memory recovery, VER-155008 or vehicle solution was intraperitoneally administered to 5XFAD mice for 18 days. Axons regrowth in the adult mouse brain takes at least 7 days after injury (Jin et al., 2016). Our previous study indicated that synaptic maturation after axonal growth required at least another 14 days (Tohda et al., 2006). We hypothesized that VER-155008 could stimulate axonal regeneration *in vivo* and thus improve memory. For expecting the axonal regeneration and subsequent synapse formation in the brain, we firstly tried to evaluate the effect VER-155008 on memory improvement at 14–18 days after administration. On day 18, a locomotion test was performed on each mouse. The total distance moved and total immobility time were not significantly different between transgenic mice treated with VER-155008 or vehicle or between either of these groups and wild-type mice treated with vehicle (**Figures 2A,B**). In addition, no significant changes in body weight were observed in any of the groups during drug administration (**Figure 2C**). These results indicate that VER-155008 treatment did not significantly affect general health and behavior.

**FIGURE 2:** VER-155008 administration rescued memory deficits in 5XFAD mice. **(A–D)** Wild-type and 5XFAD mice (female, 32–38 weeks old) were treated with VER-155008 (VER; 10 μmol/kg/day, i.p.) or vehicle solution (Veh; 10% DMSO in saline) for 18 days. **(A,B)** On administration day 18, a locomotion test was performed. Total distance moved (cm) and total immobility time (s) were measured. The differences were not significant vs. 5XFAD/Veh, one-way ANOVA *post hoc* Dunnett’s test, *n* = 4. **(C)** Change in body weight during the drug administrations (±g compared with day 0). A significant drug × day interaction was found by repeated-measures two-way ANOVA [*F*(34,153) = 1.420, *p* = 0.0788, *n* = 4]. **(D)** On administration day 14, an object recognition memory test was performed. The preferential indexes in the training and test sessions are shown. A significant drug × test interaction was found by repeated measures two-way ANOVA [*F*(2,9) = 4.230, *p* = 0.0507; ^∗^*p* < 0.05, ^∗∗∗^*p* < 0.001, *post hoc* Bonferroni test, *n* = 4]. **(E–H)** Wild-type and 5XFAD mice (female, 24–28 weeks old) were treated with VER-155008 (10 μmol/kg/day, i.p.) or vehicle solution (10% DMSO in saline) for 15 days. **(E)** On administration day 14, an object location test was performed. The preferential indexes in the training and test sessions are shown. A significant drug × test interaction was found by repeated-measures two-way ANOVA [*F*(2,12) = 35.12, *p* < 0.0001. ^∗∗∗∗^*p* < 0.0001, *post hoc* Bonferroni test, *n* = 5]. **(F)** On administration day 15, an episodic-like memory test was performed. **(G)** The preferential indexes of E_1_ + E_4_ (gray columns) and D_2_ + D_4_ (blue columns), **(H)** The preferential indexes of D_2_ (light blue columns) and D_4_ (blue columns) in the test session are shown. ^∗∗∗∗^*p* < 0.0001, unpaired *t*-test, *n* = 5.

On administration day 14, an object recognition memory test was performed. In this test, all mice showed similar exploratory behaviors toward two identical objects in the training session (preferential indexes of approximately 50%). In the test session, the VER-155008-treated 5XFAD mice showed a significantly higher preferential index to the new object did than the vehicle-treated 5XFAD mice (**Figure 2D**), indicating that VER-155008 treatment improved object recognition memory in 5XFAD mice.

To test whether spatial memory was also improved by VER-155008 administration, we performed an object location test in 5XFAD mice on administration day 14. In the test session, one of the identical objects was located in a different place compared with its location in the training session (**Figure 2E**). While wild-type mice showed higher preferential indexes for the moved object, vehicle-treated 5XFAD mice could not distinguish the two objects. However, VER-155008 administration significantly improved object location memory in the 5XFAD mice. On administration day 15, an episodic-like memory test was performed. This test requires the ability to integrate object (what), location (where), and context (when) recognition (Dere et al., 2005). Among the four objects used in test session, E_1_ and E_4_ were located at the same places in training session 2 10 min before test session (**Figure 2F**). During the test session, the objects D_2_ and D_4_ should be less familiar to the mice than objects E_1_ and E_4_. Wild-type mice showed a significantly higher preferential index for the unfamiliar (D_2_ and D_4_) than the familiar objects (E_1_ and E_4_) (**Figure 2G**). However, vehicle-treated 5XFAD mice showed equal preferential indexes to both sets of objects. VER-155008 administration increased the preferential index for the unfamiliar objects in the 5XFAD mice. Object D_2_ was placed in the test session at the same location as in training session 1, whereas D_4_ was located at a novel position compared with its location in training session 1. Therefore, mice with normal location memory should show higher preferential indexes for object D_4_ than D_2_. However, vehicle-treated 5XFAD mice failed to distinguish between D_2_ and D_4_. In contrast, VER-155008-treated mice showed significantly increased preferential indexes for D_4_, suggesting that VER-155008 administration improved episodic-like memory in the 5XFAD mice (**Figure 2H**).

Taken together, these results indicate that HSC70 inhibition ameliorated the deficits in recognition, location, and episodic-like memory in 5XFAD mice.

### VER-155008 Penetrates into the Brain after Intraperitoneal Administration in Mice

To evaluate the possibility that VER-155008 could stimulate the brain directly, we investigated whether VER-155008 crossed the BBB. By detecting the high-accuracy quasi-molecular ion ([M+H]^+^) with a mass error of ±10 mmu, we could identify the standard mass data and fragmentation pattern of VER-155008 (**Figure 3A**). Usually, doses much higher than the effective dose are used to detect compounds in biological samples by mass spectrometry (Durairajan et al., 2012; Yang et al., 2017); therefore, we administered a dose approximately 9 times higher than the dose of VER-155008 (89.9 μmol/kg) used in the experiments shown in **Figure 2** (10 μmol/kg) to 5XFAD mice. We compared extracted ion current (EIC) chromatograms of VER-155008 in plasma and cortex samples obtained from vehicle- or VER-155008-treated 5XFAD mice. In both samples from both groups of mice, total ion current peaks were detected at retention times similar to that of VER-155008 standard (**Figure 3B**). MS-MS fragmentation patterns of the peaks were also similar to that of the standard. A corresponding ion peak was not detected in the plasma and cerebral cortex of vehicle-treated mice. These results suggest that VER-155008 penetrated the BBB and reached the brain. Using a VER-155008 standard curve, the predicted concentrations of VER-15008 in the plasma and cerebral cortex were quantified as 13.97 nmol/ml and 3.326 nmol/g, respectively.

**FIGURE 3:** VER-155008 penetrates into the brain after intraperitoneal administration in 5XFAD mice. **(A)** Standard peaks of VER-155008 (1 μg/ml). Extracted ion current (EIC) chromatogram and mass spectrum (MS) of VER-155008 (m/z = 556.1246) are shown (top and bottom panels, respectively.) **(B)** 5XFAD mice (female, 36 weeks old) were treated with VER-155008 (89.9 μmol/kg/day, i.p.) or vehicle solution (10% DMSO in saline). Five min after drug administration, plasma and cortex samples were obtained. EIC chromatograms and MS graphs show the contained VER-155008 present in the biosamples.

### VER-155008 Reduced AD Pathologies in the 5XFAD Mouse Brain

After behavioral testing of drug-treated mice, we also examined the effects of VER-155008 administration on the AD-like pathological changes in 5XFAD mouse brains.

As shown in **Figure 1**, VER-155008 reversed Aβ-induced axonal atrophy in cultured neurons. Therefore we examined the effect of VER-155008 on abnormal axonal structures in the 5XFAD mouse brain. In AD patient brains, ring- or bulb-like deformed neurofilaments were located within the amyloid plaques (Dickson and Vickers, 2001). Similarly, we observed pNF-H-positive abnormal bulb-like swollen axons in the amyloid plaques in 5XFAD mice (Tohda et al., 2012). In the present study, the swollen axon area within the plaques in the perirhinal cortex or hippocampal CA1 was quantified (**Figure 4**). In wild-type mice, no deposition of amyloid plaques was observed, and the axons had fiber-like shapes. However, in the vehicle-treated 5XFAD group, the axons in the amyloid plaques were swollen. In contrast, in VER-155008-treated 5XFAD mice, the percentage of swollen axons within each amyloid plaque was reduced both in the perirhinal cortex and CA1.

**FIGURE 4:** VER-155008 administration reduced axonal swelling associated with amyloid plaques in 5XFAD mice. Wild-type and 5XFAD mice (female, 32–38 weeks old) were treated with VER-155008 (VER; 10 μmol/kg/day, i.p.) or vehicle solution (Veh; 10% DMSO in saline) for 18 days. After behavioral tests, the mice were sacrificed, and the perirhinal cortex and hippocampal CA1 were immunostained for Aβ_1-40/42_ and phosphorylated neurofilament heavy subunit (pNF-H). **(A)** pNF-H-positive and bulb-like abnormal axonal structures were localized only within the amyloid plaques. Representative images of Aβ_1-40/42_-positive amyloid plaques, pNF-H-positive axons, and DAPI staining in the perirhinal cortex are shown. The amyloid plaques area is encircled with white dotted lines. **(B)** The total area of the abnormal axons per 100 mm^2^ of amyloid plaque was quantified. ^∗∗^*p* < 0.01, ^∗∗∗^*p* < 0.001 vs. 5XFAD/Veh, one-way ANOVA *post hoc* Dunnett’s test, *n* = 4.

To investigate the effect of VER-155008 administration on the accumulation of amyloid plaques *in vivo*, the amyloid plaque areas in the perirhinal cortex and CA1 were measured (**Figure 5**). While no amyloid deposition was found in wild-type brains, the brains of age-matched vehicle-treated 5XFAD mice showed severe plaque deposition. However, the VER-155008-treated 5XFAD mice had significantly reduced total plaque areas in the perirhinal cortices and CA1 regions.

**FIGURE 5:** VER-155008 administration reduced amyloid plaques in 5XFAD mice. Aβ_1-40/42_ was visualized by immunostaining in the perirhinal cortex and hippocampal CA1. **(A)** Representative images of Aβ_1-40/42_-positive amyloid plaques in the perirhinal cortex are shown. The amyloid plaques are indicated with white arrowheads. **(B)** The total Aβ_1-40/42_-positive amyloid plaque area per 100 mm^2^ was quantified. ^∗∗∗^*p* < 0.001 vs. 5XFAD/Veh, one-way ANOVA *post hoc* Dunnett’s test, *n* = 4.

We also examined the effect of VER-155008 on the expression levels of PHF-tau (**Figure 6**). We have previously detected increased AT8-positive PHF-tau staining closely associated with amyloid plaques in 5XFAD mouse brains (Tohda et al., 2012; Yang et al., 2017). In addition, AT8-positive PHF-tau was present in 5XFAD brain lysates (Stygelbout et al., 2014). Therefore, we evaluated the AT8-positive PHF-tau levels in 5XFAD brains. While no PHF-tau was observed in wild-type mice, high PHF-tau levels were present in 5XFAD brains. The PHF-tau protein was closely associated with the amyloid plaques. Treatment with VER-155008 resulted in significant reduction of PHF-tau within the plaques in the perirhinal cortices and CA1 regions of the 5XFAD mice.

**FIGURE 6:** VER-155008 administration reduced PHF-tau associated with amyloid plaques in 5XFAD mice. Double-immunostaining for Aβ_1-40/42_ and PHF-tau was performed in the perirhinal cortex and hippocampal CA1. **(A)** Representative images of Aβ_1-40/42_-positive amyloid plaques, PHF-tau, and DAPI staining in the perirhinal cortex are shown. The amyloid plaques area is encircled with white dotted lines. **(B)** The total area of PHF-tau staining per 100 mm^2^ of amyloid plaque was quantified. ^∗∗∗^*p* < 0.001 vs. 5XFAD/Veh, one-way ANOVA *post hoc* Dunnett’s test, *n* = 4.

These results suggest that HSC70 activity is required for sustained axonal degeneration, amyloid deposition, and tau hyperphosphorylation in the brains of 5XFAD mice.

## Discussion

VER-155008, an inhibitor of HSC70, promoted axonal regrowth in cultured neurons even after axonal degeneration induced by Aβ treatment (**Figure 1**). In addition, object recognition, location, and episodic-like memory tests showed remarkable improvements in VER-155008-treated 5XFAD mice (**Figure 2**). VER-155008 penetrated the brain after intraperitoneal administration (**Figure 3**), indicating that it might affect impaired neurons directly. Axonal swelling, amyloid deposition, and PHF-tau formation were significantly reduced in the perirhinal cortices and hippocampal CA1 regions of VER-155008-treated 5XFAD mice (**Figures 4–6**). Altogether, these results suggest that VER-155008 can reverse axonal degeneration in the brain and reduce the pathological features of AD. This is the first report to demonstrate that HSC70 inhibition is sufficient to ameliorate axonal atrophy and memory dysfunction in an animal model of AD.

As a molecular chaperone, HSC70 has various client proteins, and its downstream signaling depends on which protein it associates with. The activity of HSC70 is ADP/ATP-dependent. When HSC70 has ATP in its N-terminal nucleotide-binding domain (NBD), it can associate with clients with low affinities. Through interaction with co-chaperones, the HSC70-bound ATP is hydrolyzed to give rise to an ADP-bound HSC70 with a high affinity for client proteins (Stricher et al., 2013). VER-155008 directly binds to the ATP-binding pocket of HSC70, blocking the HSC70 ATPase activity and likely preventing HSC70 binding to client proteins involved in AD-associated axonal degeneration and amyloid deposition. As mentioned above, HSC70 associates with NF-M and targets it for degradation by the UPS (Wang et al., 2011). HSC70 also associates with tau and maintains it in a hyperphosphorylated state in the AD environment (Jinwal et al., 2010). Therefore, NF-M and tau may mediate the axonal regrowth and PHF-tau reduction induced by HSC70 inhibition in 5XFAD brains. Our results are consistent with the findings that allosteric HSP70 inhibitors reduced tau levels and stimulated long-term potentiation in *ex vivo* brain slices from a transgenic mouse tauopathy model (Abisambra et al., 2013).

No direct evidence exists that HSC70 is related to amyloid plaque accumulation. Sp1 is transcription activator of the genes encoding beta-site amyloid precursor protein-cleaving enzyme (BACE) 1 and amyloid precursor protein (APP), abnormal processing of which causes Aβ accumulation in AD brains (Christensen et al., 2004). Sp1 expression is increased in AD patients and model mouse brains (Citron et al., 2008). Importantly, Sp1 is also a client protein of HSC70, which protects Sp1 from degradation (Yang et al., 2014). This finding indicates that HSC70 activity correlates with Sp1 upregulation, possibly leading to the accumulation of amyloid plaques. Therefore, VER-155008 may downregulate Sp1 expression and prevent amyloid plaque formation by inhibiting HSC70 activity. However, in the present study, we used 7–8-month-old 5XFAD mice, and the drug administration period was only 18 days. At this age, the accumulation of amyloid plaques in the mouse brain had almost plateaued (Oakley et al., 2006). VER-155008 treatment decreased the plaque areas in the 5XFAD brains by 50% in the perirhinal cortex and 43% in the CA1 relative to the vehicle-treated group (**Figure 5**). Therefore, we speculate that the VER-155008-induced reduction of amyloid plaques is caused not only through prevention of plaque production, but also through other effects, such as increased plaque degradation. Further investigation is required to clarify the mechanism underlying the reduction of amyloid plaques by of HSC70 inhibition.

Pharmacokinetics studies of VER-155008 showed that VER-155008 penetrated into tumor tissues after intravenous administration (Massey et al., 2010). However, no reports have focused on BBB penetration by VER-155008. The hydrophobicity of VER-155008 is comparatively high (Clog *P* = 2.71). **Figure 3** indicates that VER-155008 reached the brain. Moreover, we found that several pathological features (swollen axons, amyloid plaques, and PHF-tau levels) in the brain were reduced by VER-155008 administration (**Figures 4–6**), suggesting that VER-155008 acts in the brain. During VER-155008 administration, no significant changes in body weight or abnormal behavior were observed (**Figures 2A–C**), suggesting that administration of VER-155008 is safe and effective, at least at the dose used in this study.

This is the first report to show that HSC70 inhibition effectively reverses axonal degeneration and recovers memory function in AD-like pathologies. Fortunately, several HSC70 inhibitors have recently been developed. However, these inhibitors, including VER-155008, were created to treat cancer because HSC70 activates autophagy pathways and inhibits apoptosis for the survival of cancer cells (Liu et al., 2012). In the present study, we utilized these properties of VER-155008 to stimulate axonal regrowth and memory recovery. HSC70 may be a new, promising therapeutic target for the treatment of AD and other neurodegenerative diseases.

## Author Contributions

XY and CT designed the experiments and drafted the manuscript. XY performed the experiments and analyzed the data. CT supervised all the experiments and analyses.

## Conflict of Interest Statement

The authors declare that the research was conducted in the absence of any commercial or financial relationships that could be construed as a potential conflict of interest.
